# M2 Macrophage-Derived Exosomes Inhibit Apoptosis of HUVEC Cell through Regulating miR-221-3p Expression

**DOI:** 10.1155/2022/1609244

**Published:** 2022-09-07

**Authors:** Xiandong Cheng, Hong Zhou, Ying Zhou, Cheng Song

**Affiliations:** Department of Pulmonary and Critical Care Medicine, The Central Hospital of Wuhan, Tongji Medical College, Huazhong University of Science and Technology, Wuhan 430014, China

## Abstract

Atherosclerosis (AS) is associated with high morbidity and mortality rates and currently has no effective treatment. This study was aimed at investigating the role of macrophage exosomes in the inflammation and apoptosis after HUVEC injury. We established the HUVEC injury model using 100 mg/L oxidized low-density lipoprotein (ox-LDL) or 50 ng/mL tumor necrosis factor-*α* (TNF-*α*). Cell proliferation was assessed using cell counting kit-8 (CCK8) assays, and the expression of miR-221, TNF-*α*, and IL-6, IL-10, and IL-1*β* was detected using quantitative real-time PCR (qRT-PCR). The apoptotic rate was analyzed by the TUNEL method, and the expressions of apoptosis-related proteins Bcl2, Caspase-3, and c-myc were detected by western blotting. Finally, miR-221-3p mimics and miR-221-3p inhibitors were constructed by liposome transfection to determine the mechanism of action of macrophage exosomes on HUVEC injury. The expression levels of IL-6, IL-1*β*, and TNF-*α* in the injury groups were higher than those in the normal group, but the expression of IL-10 in the injury groups was lower than that in the normal group. Meanwhile, the apoptotic rate of the HUVEC cell injury group was higher than that of the normal group. In contrast, the expression levels of IL-6, IL-1*β*, and TNF-*α* were lower in the M2 macrophage exosome (M2-Exo) group, but the expression of IL-10 was higher compared with the control group. The apoptosis rate was reduced in the M2-Exo group, and the expression of the proapoptotic gene Caspase-3 was reduced, while the expression of the antiapoptotic gene Bcl2 was increased. Liposome transfection of miR-221-3p mimics was able to enhance the effect of M2 macrophage exosomes. Thus, M2-Exo promotes HUVEC cell proliferation and inhibits HUVEC cell inflammation and apoptosis. miR-221-3p overexpression attenuates HUVEC cell injury-induced inflammatory response and apoptosis, while miR-221-3p gene inhibition enhances this inflammatory response and apoptosis.

## 1. Introduction

Atherosclerosis (AS) is a multifactorial chronic inflammatory disease that commonly leads to cardiovascular disease [1]. The pathogenesis of AS predominantly involves dysfunction of vascular endothelial cells leading to release of the MCP-1/CCR2 complex and subsequent recruitment of monocytes into the intimal polarization of arteries. This leads to the formation of macrophages, which phagocytose lipid substances to form foam cells, which subsequently accumulate and form atherosclerotic plaques. The development of atherosclerosis involves many cells, such as endothelial cells, vascular smooth muscle cells, and macrophages. One of the most important factors appears to be the function and relative ratio of different macrophage phenotypes [1]. Changes in plaque size and stability are predominantly due to macrophage polarization. The main drugs currently used for clinical treatment of AS are statins, whose main mechanism of action is to reduce lipid concentrations [2]. However, novel treatment strategies for AS have been proposed, including decreasing the local proliferation of proinflammatory macrophage subpopulation or enhancing the regression of inflammation [3]. Therefore, modifying the regulation of macrophage activity could be effective in the treatment of atherosclerosis. However, the mechanism of action of different macrophage phenotypes on AS development remains unclear.

Lee et al. investigated the characteristics and phenotypic changes of macrophages in AS and the effect of cytoplasmic lipid accumulation on the macrophage phenotype. It was demonstrated that the inflammatory phenotype triggered by oxidized low-density lipoprotein (ox-LDL) downregulates the activation of anti-inflammatory genes, leading to tissue repair [4]. It has been shown that macrophages differ in phenotype and function in various stages of atherosclerosis [5]. Macrophages can be divided into two types, M1 and M2 macrophages. M1 macrophages can be polarized by IFN-*γ* and LPS and have a proinflammatory function. They are capable of secreting inflammatory factors such as MCP-1, IL-12, IL-23, and tumor necrosis factor-*α* (TNF-*α*) and activate oxidative stress and apoptotic pathways. M2 macrophages have anti-inflammatory effects and can induce polarization through IL-4 and IL-13. They secrete anti-inflammatory factors such as IL-10, TGF-*β*, YM-1, arginase I, and chemokines [6, 7]. M1 macrophages can be converted to M2 macrophages in the presence of high anaerobic glycolysis, fatty acid synthesis, and a shortened citric acid cycle. Sufficient IL-4 is essential for the maintenance of M2 macrophages, which will convert back to the M1 phenotype if IL-4 is deficient [8]. Zheng et al. discovered that miR-155 can inhibit tight junction protein expression and damage endothelial cells (ECs). It was also shown that miR-155 inhibits EC proliferation and migration, resulting in tissue damage [9]. Therefore, we speculated that macrophage-mediated damage of human umbilical vein edothelial cells (HUVECs) might be mediated by exosomes (Exos, which contain miRs), and aimed to elucidate the specific mechanism of action.

Exos are bilayer nanovesicles secreted by cells that deliver lipids, proteins, and nucleic acids to other cells to regulate various pathways [10]. Macrophage Exos can attenuate the inflammatory response of recipient cells by regulating cytokines and miRNA levels [11]. It has been demonstrated that Exos exert anti-inflammatory effects by inhibiting the secretion of proinflammatory enzymes and cytokines and induces HUVEC cell proliferation and migration to accelerate the wound healing process, thereby improving angiogenesis and epithelial reformation in diabetic wounds [12]. It has been shown that proinflammatory M1 macrophages release large amounts of proinflammatory exosomes (M1-Exos) that inhibited the Sirt1/AMPK*α*2-endothelial-type nitric oxide synthase and RAC1-PAK2 signaling pathways by simultaneously targeting five molecular nodes (genes) to reduce the angiogenic capacity of HUVECs [13]. However, the role and potential mechanisms of macrophages in atherosclerotic angiogenesis and injury repair remain unclear.

The aim of this study was to investigate the mechanisms underlying the effects of macrophage-Exo miRNA on HUVEC injury in atherosclerosis. Six miRNAs were screened using bioinformatics methods: hsa-miR-4449, hsa-miR-211-5p, hsa-miR-10b-3p, hsa-miR-503-5p, hsa-miR-708-5p, and hsa-miR-221-3p. We induced macrophage polarization in vitro, examined the expression of miRNA in macrophages, and examined their Exos *in vitro*. Meanwhile, a HUVEC injury model was established, and the mechanism of HUVEC injury by macrophage-Exo miRNA through its target Grb10 was investigated. This provides an important theoretical basis for the subsequent study of the mechanism of HUVEC injury.

## 2. Materials and Methods

### 2.1. Cell Culture and Transfection

Human monocytic leukemia cells (THP-1) and human umbilical vascular endothelial cells (HUVECs) were purchased from the Shanghai Cell Bank of the Chinese Academy of Sciences. THP-1 cells were cultured in BPMI 1640 medium (TBD, Tianjin, China) with 10% fetal bovine serum (Procell, Wuhan, China), and HUVECs were cultured in a primary HUVEC cell culture system (iCell, Shanghai, China) with 10% fetal bovine serum. The cells were maintained at 37°C with 5% CO_2_. HUVECs (5 × 10^5^/well) were seeded in a 6-well plate and incubated for 24 h for integration. The cells were then transfected with Opti-MEM (Sigma, USA) and Lipofectamine® RNAiMAX (Life Technologies, Shanghai, China) according to the manufacturer's instructions. The expression of miR-221-3p was detected at 48 h posttransfection.

### 2.2. Macrophage Polarization

THP-1 cells were inoculated in RPMI 1640 medium at 37°C with 5% CO_2_ and constant 60%-70% humidity in an incubator. Cells were then cultured with 5 × 10^6^ cells/well in a 12-well plate and induced by PMA (Sigma, USA) at a concentration of 100 *μ*g/L for 48 h. After the cells changed from the suspended to the adherent, they were washed twice with PBS and the culture medium was changed.

The induced cells were divided into 3 groups: M0, M1, and M2 groups. No reagents were added to the M0 group, 100 *μ*g/L lipopolysaccharide (LPS) and 20 *μ*g/L IFN-*γ* were added to the M1 group, and 20 *μ*g/L IL-4 was added to the M2 group for 24 h. The cell morphology of each group was observed using light microscopy (Shanghai Ruixian Biotechnology Co.).

### 2.3. Isolation of Exosomes

Macrophages were cultured in RPMI 1640 medium (ultracentrifuged at 120,000 g for 16 h) with 10% FBS for 24 h. The cell-conditioned medium was centrifugated at 15,000 rpm for 3 min, followed by filtration through a 0.22 *μ*m filter. Next, the supernatant was removed by ultracentrifugation at 57,000 rpm for 1 h, and the clear precipitate at the bottom of the centrifuge tube (containing the Exos) was collected, which was the exosome (Exo) of macrophages. Finally, 10 *μ*g of Exo was resuspended in 100 *μ*L PBS.

### 2.4. Transmission Electron Microscopy

Isolated Exos were fixed with 4% paraformaldehyde and added to the copper mesh. Then, Exos were fixed with 1% glutaraldehyde for 20 min. Samples were stained with uranium acetate for 5 min in the absence of light and then washed with double-distilled water. The samples were blotted dry on filter paper, observed using transmission electron microscopy, and photographed (Hitachi, HT7700).

### 2.5. Real-Time Quantitative PCR

Total RNA was extracted from cells or Exo using TRIzol (Ambion, USA). RNA was then reverse transcribed to cDNA using PrimeScript II RTase (TAKARA, Japan). The cDNA was amplified using SYBR FAST qPCR Master Mix (KAPA biosystems). Reaction conditions were 40 cycles of 95°C for 3 min, 95°C for 5 s, and then 56°C for 10 s followed by 72°C for 25 s. The primer sequences are listed in Table 1. GAPDH and U6 gene were used as the housekeeping gene. The mRNA was calculated using the 2^-*ΔΔ*t^ method.

### 2.6. Western Blotting

Cells or Exos were isolated and denatured in RIPA buffer (Ambion, USA) for total protein. Total protein (20 *μ*g) was separated by sodium dodecyl sulfate-polyacrylamide gel electrophoresis (SDS-PAGE) gel and transferred onto PVDF membranes (DOCLAB, Korea). Membranes were blocked in 5% nonfat milk for 1 h, then incubated overnight at 4°C with primary antibodies (all from bioswamp, at 1 : 1000 dilution), including anti-IL-12, anti-Arg1, anti-iNOS, anti-CD206, anti-Caspase-3, anti-Bcl2, anti-c-myc, anti-Grb10, and anti-GAPDH antibodies, followed by incubation with secondary antibodies anti-Rabbit IgG (bioswamp, 1 : 20000 dilution) for 1 h at 25 ± 2°C, and visualization using the ECL chemiluminescence reagent (Beyotime, Jiangsu, China).

### 2.7. Establishment of HUVEC Cell Injury Model

The vascular HUVEC cell oxidative stress injury model was established by inoculating HUVECs in 12-well plates with 100 mg/L oxidized low-density lipoprotein (ox-LDL) in culture medium for 24 h (control group). Macrophages were cocultured with HUVECs. The numbers of macrophages and endothelial cells in the 24-well plate used in the cell counting kit-8 (CCK8) experiment were 4 × 10^4^ and 1.2 × 10^5^, respectively, while the numbers of macrophages and endothelial cells in the 6-well plate used in other experiments were 2 × 10^5^ and 6 × 10^5^, respectively (M0, M1, and M2 groups). The apoptosis of cells was detected by flow cytometry, and proliferation was measured by CCK8 assay. HUVECs were used as the normal group.

In the vascular HUVEC inflammatory injury model, HUVECs were cultured in 12-well plates with 50 ng/mL TNF-*α* in the medium for 24 h (control group). Apoptosis was tested by flow cytometry, and proliferation was detected by CCK8 assay. HUVECs were used as the normal group.

### 2.8. Cell Counting Kit-8 Assay

Cell proliferation was measured using the cell counting kit-8 (CCK8) (Bioswamp, USA). HUVECs (3 × 10^3^/well) were seeded into a 96-well plate, and 10 *μ*L CCK8 reagent was added to each well at the time of harvest. Next, the HUVECs were cultured at 37°C for 1 h. Finally, the absorbance at 450 nm (OD_450nm_) was measured to determine the cell viability using a microplate reader (SpectraMax, USA). The data were representative of three independent experiments performed in triplicate.

### 2.9. TUNEL Assay

Cells were harvested by centrifugation at 1500 rpm for 5 min and washed with PBS for 3 times, and apoptosis was measured using the Annexin V-FITC/PI Apoptosis Assay Kit. Stained cells were detected using a Quanteon flow cytometer (Agilent, California, USA).

### 2.10. Statistical Analysis

Data were presented as the mean ± SD, and graphs were generated with GraphPad Prism 5.0. Statistical analysis between multiple groups was performed using one-way analysis of variance (ANOVA). Differences were considered statistically significant at *P* value < 0.05.

## 3. Results

### 3.1. Phenotype and Characterization of Induced Macrophage Polarization In Vitro

Previous studies have shown that PMA can induce the differentiation of THP-1 cells into macrophages [14]. To explore the influence of macrophages on HUVEC cell injury, we induced the differentiation of THP-1 cells into macrophages and polarized macrophages into M1 and M2 macrophages. Observation under an optical microscope revealed that the macrophages changed from suspended to adnate growth and from round to irregular in shape (Figure 1(a)). The M1 and M2 macrophages were also characterized by western blot analysis, to evaluate the expression of specific markers, including iNOS, IL-12, and Arg1, as well as CD206 (Figures 1(b) and 1(c)). The results showed that M1 macrophages displayed high iNOS and IL-12 protein expression, whereas M2 macrophages displayed high Arg1 and CD206 protein expression.

### 3.2. Extraction and Identification of M0, M1, and M2 Macrophage Exosomes

To demonstrate the mechanism of Exo on HUVEC cell injury, we isolated cell-derived Exos from the supernatant of M0, M1, and M2 macrophages. Under a transmission electron microscope (Figure 2(a)), Exos displayed a complete structure in the shape of round vesicles. Western blotting results (Figures 2(b) and 2(c)) showed that the secretion-specific biomarkers Alix, CD63, and Tsg101 were positive in M0, M1, and M2 macrophages, respectively, suggesting the successful extraction of M0, M1, and M2 macrophages.

### 3.3. Model Construction and Identification

To elucidate the effects of macrophages and Exos on HUVEC cell injury, we then constructed a HUVEC cell oxidative stress injury model and a HUVEC cell inflammatory injury model. CCK8 assays showed that cell proliferation was significantly lower in the oxidative stress group than in the normal group. Flow cytometry analysis showed that the percentage of apoptotic cells was significantly higher in the oxidative stress injury group than in the normal group (Figure 3(a)). The results of the HUVEC inflammatory injury model were consistent with those in the HUVEC oxidative stress injury model (Figure 3(b)).

### 3.4. Effects of the M0, M1, and M2 Macrophage Phenotypes on HUVEC Cell Injury

We next tested whether macrophages affect the proliferation and apoptosis of HUVECs by coculturing macrophage with HUVECs. In the HUVEC cell oxidative stress injury model, CCK8 assays showed that M2 macrophages significantly enhanced HUVEC proliferation compared to the control group (Figure 4(b)). Flow cytometry analysis showed that the percentage of apoptotic cells was significantly decreased in the M2 group than in the control group (Figures 4(a) and 4(c)). Furthermore, qRT-PCR results demonstrated that M2 macrophages markedly reduced the expression of IL-6, IL-1*β*, and TNF-*α*, while increasing the expression of IL-10 (Figure 4(d)). Moreover, western blotting results showed that M2 macrophages increased the protein levels of Bcl2 and c-myc and reduced those of cleaved-Caspase-3 (Figure 4(e)). We also tested the effect of macrophages in the HUVEC cell inflammatory injury model. These results were consistent with those in the HUVEC cell oxidative stress injury model (Figure 5).

### 3.5. Effects of the M0, M1, and M2 Macrophage Exosomes on HUVEC Cell Injury

Next, we tested whether macrophage Exos affected the proliferation and apoptosis of HUVECs. In the HUVEC cell oxidative stress injury model (Figure 6(b)), M2 macrophage Exos significantly restored HUVEC cell proliferation. Flow cytometry analysis showed that the percentage of apoptotic cells was significantly decreased in the M2 group (Figures 6(a) and 6(c)). Moreover, M2 macrophage exos significantly reduced the expression of IL-6, IL-1*β*, and TNF-*α*, while increasing the expression of IL-10 (Figure 6(d)). Western blotting results showed that M2 exos increased the protein levels of Bcl2 and c-myc and reduced the protein levels of cleaved-Caspase-3 (Figure 6(e)). The results in the HUVEC inflammatory injury model were consistent with those in the HUVEC cell oxidative stress injury model (Figure 7).

### 3.6. Exosomes Affect HUVEC Cell Injury via the miR-221-3p/Grb10 Axis

To investigate the miRNAs involved in the mechanism of macrophage and Exo-induced restoration of HUVEC cell injury, the miRNA expression of miR-4449, miR-211-5p, miR-10b-3p, miR-503-5p, miR-708-5p, and miR-221-3p was detected. We found that miR-221-3p displayed the most abundant expression in M2 macrophages and macrophage Exos (Figure 8(a)). The qRT-PCR experiment revealed the highest miR-221-3p expression in the miR-221-3p mimics group and the lowest miR-221-3p expression in the miR-221-3p inhibitor group, confirming that the transfection was successful (Figure 8(b)). Moreover, in the HUVEC oxidative stress injury model (Figure 8(d)), miR-221-3p mimics significantly restored HUVEC cell proliferation, but miR-221-3p inhibitors significantly inhibited cell proliferation. Flow cytometry analysis showed that the percentage of apoptotic cells was significantly decreased in the miR-221-3p mimics group and increased in the miR-221-3p inhibitor group (Figures 8(c) and 8(e)). qRT-PCR results showed that miR-221-3p mimics significantly reduced the expression of IL-6, IL-1*β*, and TNF-*α* but increased the expression of IL-10 (Figure 8(f)). Meanwhile, miR-221-3p mimics increased the protein levels of Bcl2 and c-myc and reduced the protein levels of Caspase-3 and Grb10 (Figure 8(g)). The results in the HUVEC inflammatory injury model were consistent with those in the HUVEC oxidative stress injury model (Figure 9).

## 4. Discussion

Due to the key role of macrophages in AS, macrophages are first recruited to the endothelium and transformed into foam cells, which secrete various substances that affect neighboring cells, such as HUVECs and macrophages during all stages of AS [15]. HUVEC dysfunction and morphological damage can manifest as multiple physiological effects, including adhesion of leukocytes, vasoconstriction, platelet activation, oxidative stress, and inflammation, which ultimately lead to the development of AS. Therefore, promoting HUVEC proliferation, inhibiting HUVEC apoptosis, and suppressing HUVEC inflammation have become key strategies for the prevention and control of AS [9, 16]. Undoubtedly, macrophages are the primary concern in the treatment of HUVEC cell injury.

Exos are nanosized extracellular vesicles released by a variety of cells which contain small noncoding RNAs, such as miRNAs, proteins, and lipids. The bilayer lipid-like membrane of Exos protects these contents from degradation and allows intercellular communication [17]. Oxidative low-density lipoprotein- (ox-LDL-) induced oxidative stress and TNF-*α*-induced cellular inflammation are key to AS development. It has been shown that the role of lncRNA Gas5 in the formation of AS is to regulate apoptosis of macrophages and HUVECs through Exos, suggesting that inhibition of lncRNA Gas5 may be an effective way to treat AS [18]. Zhou et al. suggested that ginsenoside Rb1 protects HUVECs from TNF-*α*-induced oxidative stress and inflammatory responses by inhibiting the action of JNK and p38 [19]. In our study, Exos secreted by macrophages were identified using electron microscopy and protein blotting. We next established an HUVEC cell injury model using induction by oxidized low-density lipoprotein (ox-LDL) and TNF-*α*, which showed that M2 macrophages and M2 macrophage Exos promoted HUVEC cell proliferation while inhibiting HUVEC cell apoptosis and inflammatory responses. However, the exact mechanism of action remains unclear.

Recently, miRNA expression in various diseases has been extensively studied, but its functions and regulatory mechanisms have not been fully explored. Dysregulation of miRNAs is associated with the progression of various diseases, affecting cell proliferation, apoptosis, and migration [20–22]. There is evidence that the Exos of MSCs can transfer miRNAs to HUVECs and promote angiogenesis [23].

Meanwhile, we screened six miRNAs by bioinformatics methods, including hsa-miR-4449, hsa-miR-211-5p, hsa-miR-10b-3p, hsa-miR-503-5p, hsa-miR-708-5p, and hsa-miR-221-3p. qRT-PT results showed that the miR-221-3p expression was increased in M2 macrophage Exos. Previous studies have uncovered a role for miR-221 in a variety of cancers. miR-221 has been reported to play a cancer-promoting role in breast cancer [24] and nonsmall cell lung cancer [25], whereas it plays a cancer-inhibiting role in laryngeal cancer [26]. However, there are relatively few studies on the effects of miR-221-3p on HUVEC cell injury. Recent studies have shown that the OGD-induced inflammatory response and apoptosis are attenuated by miR-221 overexpression and enhanced by miR-221 knockdown [27]. It has also been found that miR-221 attenuates brain injury during acute ischemic stroke by inhibiting the proinflammatory response [28].

In this study, we investigated the mechanism of miR-221-3p involvement in the treatment of HUVEC cell injury by macrophage Exos. We transfected miR-221-3p mimics and miR-221-3p inhibitors by liposome and then applied macrophage Exos to HUVECs. The results showed that macrophage Exos transfected with miR-221-3p mimics promoted HUVEC cell proliferation, but inhibited HUVEC cell apoptosis and HUVEC cell inflammatory responses, which is consistent with previous studies. Previous studies have also shown that NGR1 inhibits TLR 4/NF-*κ*B pathway activation by increasing the miR-221-3p expression and reducing OX-LDL-induced apoptosis, inflammation, and oxidative stress in HUVECs [29]. Therefore, our results are consistent with those of previous studies. As we measured a decrease in Grb10 expression, we speculate that miR-221-3p may act by targeting Grb10, but further experiments are needed to confirm this.

Overall, M2 MSC-Exos exerted a therapeutic effect on HUVEC cell injury by promoting HUVEC cell proliferation and inhibiting HUVEC cell apoptosis and inflammation, while suppressing Grb10 expression, providing a promising therapeutic modality for AS.

## Figures and Tables

**Figure 1:** Characterization of M0, M1, and M2 macrophages. (a) M0, M1, and M2 macrophages were induced by 100 *μ*g/L PMA for 48 h, and the cellular morphology was observed under a light microscope, scale bar: 50 *μ*m (*n* = 1). (b) Macrophages were identified by western blotting using anti-iNOS, anti-IL-12, anti-Arg1, and anti-CD206 antibodies (*n* = 3). (c) Levels of iNOS, IL-12, Arg1, and CD206 protein expression in macrophages. ^∗^Compared with M0 group; ^∗∗∗^*P* < 0.001; ^#^compared with M2 group; ^###^*P* < 0.001.

**Figure 2:** Macrophage-derived exosome characterization. (a) Exosomes were isolated from M0, M1, and M2 macrophages, and the morphology and size were confirmed by transmission electron microscopy, scale bar: 200 nm (*n* = 1). (b) Macrophage-derived exosomes were analyzed by western blotting using anti-Alix, anti-CD63, and anti-Tsg101 antibodies (*n* = 3). (c) Levels of Alix, CD63, and Tsg101 protein expression in macrophage-derived exosomes. ^∗^Compared with M0 group; ^∗∗∗^*P* < 0.001; ^#^compared with M2 group; ^###^*P* < 0.001.

**Figure 3:** Construction of HUVEC oxidative stress and inflammatory injury models. A: HUVECs were cultured with 100 mg/L oxidized low-density lipoprotein (ox-LDL) for 24 h to establish an oxidative stress injury model. Cell proliferation was detected by CCK8 assays, and cell apoptosis was determined using Annexin V-FITC/PI staining followed by flow cytometry (*n* = 3). B: HUVECs were cultured with 50 ng/mL tumor necrosis factor-*α* (TNF-*α*) for 24 h to establish an inflammatory injury model, Cell proliferation was measured by CCK8 assay, and cell apoptosis assay was determined with Annexin V-FITC/PI staining followed by flow cytometry analysis (*n* = 3). ^∗^compared with Normal group; ^∗∗∗^*P* < 0.001.

**Figure 4:** M2 macrophages enhanced HUVEC cell proliferation and inhibited HUVEC cell apoptosis in the HUVEC oxidative stress injury model. (a, c) Cell apoptosis assays were performed using Annexin V-FITC/PI staining followed by flow cytometry (*n* = 3). (b) Cell proliferation was determined using CCK8 assays. HUVECs were treated with or without M0, M1, or M2 macrophages (*n* = 3). (d) qRT-PCR analysis of mRNA levels of inflammatory factors IL-6, IL-10, IL-1*β*, and TNF-*α* mRNA in HUVECs (*n* = 3). (e) Representative western blots of apoptosis-related protein (Caspase-3, Bcl2, and c-myc) expressions in HUVECs after macrophage stimulation (*n* = 3). ^∗^Compared with control group. ^∗^*P* < 0.05, ^∗∗^*P* < 0.01, ^∗∗∗^*P* < 0.001.

**Figure 5:** M2 macrophages enhanced HUVEC proliferation and inhibited HUVEC cell apoptosis in the HUVEC inflammatory injury model. (a, c) Cell apoptosis assay was determined using Annexin V-FITC/PI staining followed by flow cytometry (*n* = 3). (b) Cell proliferation was determined using CCK8 assays. HUVECs were treated with or without M0, M1, or M2 macrophages (*n* = 3). (d) qRT-PCR analyses of mRNA levels of inflammatory factors IL-6, IL-10, IL-1*β*, and TNF-*α* in HUVECs (*n* = 3). (e) Representative western blots of apoptosis-related protein (Caspase-3, Bcl2, and c-myc) expressions in HUVEC cells after macrophage stimulation (*n* = 3). ^∗^Compared with control group. ^∗^*P* < 0.05, ^∗∗^*P* < 0.01, ^∗∗∗^*P* < 0.001.

**Figure 6:** M2 macrophage Exos enhanced HUVEC cell proliferation and inhibited HUVEC cell apoptosis in the HUVEC cell oxidative stress injury model. (a, c) Cell apoptosis assay was determined using Annexin V-FITC/PI staining followed by flow cytometry (*n* = 3). (b) Cell proliferation was determined using CCK8 assays. HUVECs were treated with or without M0, M1, or M2 macrophage Exos (*n* = 3). (d) qRT-PCR analyses of mRNA levels of inflammatory factors IL-6, IL-10, IL-1*β*, and TNF-*α* mRNA in HUVECs (*n* = 3). (e) Representative western blots of apoptosis-related protein (Caspase-3, Bcl2, and c-myc) expressions in HUVEC cells after Exos stimulation (*n* = 3). ^∗^Compared with control group. ^∗^*P* < 0.05, ^∗∗^*P* < 0.01, ^∗∗∗^*P* < 0.001.

**Figure 7:** M2 macrophage Exos enhanced HUVEC cell proliferation and inhibited HUVEC cell apoptosis in the HUVEC cell inflammatory injury model. (a, c) Cell apoptosis assay was determined using Annexin V-FITC/PI staining followed by flow cytometry (*n* = 3). (b) Cell proliferation was determined using CCK8 assay. HUVECs were treated with or without M0, M1, or M2 macrophage Exos (*n* = 3). (d) qRT-PCR analyses of inflammatory factors IL-6, IL-10, IL-1*β*, and TNF-*α* mRNA in HUVECs (*n* = 3). (e) Representative western blots of apoptosis-related protein (Caspase-3, Bcl2, and c-myc) expressions in HUVEC cells after Exos stimulation (*n* = 3). ^∗^Compared with control group. ^∗^*P* < 0.05, ^∗∗^*P* < 0.01, ^∗∗∗^*P* < 0.001.

**Figure 8:** Effect of miR-221-3p in the HUVEC oxidative stress injury model. (a) The relative miRNA expression of miR-4449, miR-211-5p, miR-10b-3p, miR-503-5p, miR-708-5p, and miR-221-3p in macrophages and macrophage Exos (*n* = 3). (b) The relative miRNA expression of miR-221-3p after transfection (*n* = 3). (c, e) Cell apoptosis assay was determined using Annexin V-FITC/PI staining followed by flow cytometry (*n* = 3). (d) Cell proliferation was determined by CCK8 assay (*n* = 3). (f) qRT-PCR analyses of inflammatory factors IL-6, IL-10, IL-1*β*, and TNF-*α* mRNA in HUVECs (*n* = 3). (g) Representative western blots of apoptosis-related proteins (Caspase-3, Bcl2, and c-myc) and Grb10 protein expression in HUVEC cells after liposome transfection (*n* = 3). ^∗^Compared with control group; ^∗^*P* < 0.05, ^∗∗^*P* < 0.01, ^∗∗∗^*P* < 0.001.

**Figure 9:** Effect of miR-221-3p in the HUVEC inflammatory injury model. (a, c) Cell apoptosis assay was determined using Annexin V/PI staining followed by flow cytometry (*n* = 3). (b) Cell proliferation was determined by CCK8 assay (*n* = 3). (d) qRT-PCR analyses of inflammatory factors IL-6, IL-10, IL-1*β*, and TNF-*α* mRNA in HUVECs (*n* = 3). (e) Representative western blots of apoptosis-related proteins (Caspase-3, Bcl2, and c-myc) and Grb10 protein expression in HUVEC cells after liposome transfection (*n* = 3). ^∗^Compared with control group. ^∗^*P* < 0.05, ^∗∗^*P* < 0.01, ^∗∗∗^*P* < 0.001.

**Table 1:** The primer sequences.

Gene name	Primer sequence
miR-4449-F	GGCGTCCCGGGGCTGC
miR-4449-R	AACTGGTGTCGTGGAGTCGGC
miR-211-5p-F	GGGGTTCCCTTTGTCATCCT
miR-211-5p-R	AACTGGTGTCGTGGAGTCGGC
miR-10b-3p-F	GGGGACAGATTCGATTCTAG
miR-10b-3p-R	AACTGGTGTCGTGGAGTCGGC
miR-503-5p-F	GGGGTAGCAGCGGGAACAG
miR-503-5p-R	AACTGGTGTCGTGGAGTCGGC
miR-708-5p-F	GGGGAAGGAGCTTACAATCTA
miR-708-5p-R	AACTGGTGTCGTGGAGTCGGC
miR-221-3p-F	GGGGAGCTACATTGTCTGCTG
miR-221-3p-R	AACTGGTGTCGTGGAGTCGGC
U6-F	CTCGCTTCGGCAGCACA
U6-R	AACGCTTCACGAATTTGCGT
IL-6-F	AGCCACTCACCTCTTCA
IL-6-R	TCTTTGCTGCTTTCACA
IL-10-F	GGAGAACCTGAAGACCCTC
IL-10-R	ACTCACTCATGGCTTTGTAGAT
IL-1*β*-F	AGTGGCAATGAGGATGA
IL-1*β*-R	GTAGTGGTGGTCGGAGA
TNF-*α*-F	CAGGCGGTGCTTGTTC
TNF-*α*-R	TGTCACTCGGGGTTCG
GAPDH-F	GGGAAACTGTGGCGTGAT
GAPDH-R	GAGTGGGTGTCGCTGTTGA

## Data Availability

Only the summary of the data has been reported in this article. On the basis of reasonable request, datasets are available from the corresponding author.
